The article "Ductal carcinoma in situ of the breast: correlation between histopathological features and age of patients" was published in 2014. Journal: Diagn Pathol.

# Ductal carcinoma in situ of the breast: correlation between histopathological features and age of patients

**DOI:** 10.1186/s13000-014-0227-3

**Published:** 2014-12-03

**Authors:** Amanda Arantes Perez, Débora Balabram, Marcio de Almeida Salles, Helenice Gobbi

**Affiliations:** Breast Pathology Laboratory, School of Medicine, Federal University of Minas Gerais, Av. Prof. Alfredo Balena, 190, Belo Horizonte, Minas Gerais, Brasil

**Keywords:** Ductal carcinoma in situ, Histological pattern, Morphology, Breast cancer

## Abstract

**Background:**

The histopathological subtype, nuclear grade and presence or absence of comedonecrosis are established as critical elements in the reporting of ductal carcinoma in situ (DCIS) of the breast. The aims of this study were to determine the frequencies of morphological subtypes of DCIS, nuclear grade and comedonecrosis; to compare the age of patients with the histopathological characteristics of DCIS, and to assess the agreement of grade between in situ and invasive components in DCIS cases that were associated with invasive carcinoma.

**Methods:**

We evaluated a series of 403 cases of DCIS, pure or associated with invasive mammary carcinoma, consecutively identified from the histopathology files of the Breast Pathology Laboratory, Federal University of Minas Gerais, Brazil, from 2003 to 2008.

**Results:**

DCIS displayed a single growth pattern in most cases (55.1%) and the solid subtype was the most common morphology (42.2% of the total). High-grade DCIS was identified in 293/403 cases (72.7%) and comedonecrosis was present in 222/403 cases (55%). Among DCIS with a single architectural pattern, high grade was more common in the solid subtype (151/168 cases, 89.9%; p < 0.001). Only 32% of tumours with a cribriform pattern had high nuclear grade. Comedonecrosis was more common in the solid morphology than in the cribriform, papillary and micropapillary subtypes (p < 0.001). Patients with high-grade DCIS were younger in relation to patients with low-grade DCIS (p = 0.027) and patients with tumours with comedonecrosis were also younger in comparison to patients with tumours without comedonecrosis (p = 0.003). Fair agreement was observed between in situ and invasive components with regard to grade (weighted kappa = 0.23).

**Conclusions:**

The high nuclear grade and the presence of comedonecrosis were identified more frequently in younger patients and more often correlated with the solid pattern of DCIS.

**Virtual Slides:**

The virtual slide(s) for this article can be found here: http://www.diagnosticpathology.diagnomx.eu/vs/13000_2014_227

## Background

Ductal carcinoma in situ of the breast (DCIS) is defined as a neoplastic proliferation of epithelial cells confined to the mammary ductal-lobular system and characterized by subtle to marked cytological atypia and an inherent but not necessarily obligate tendency for progression to invasive breast cancer [1]. DCIS constitutes 20% of all newly diagnosed breast cancer cases and 30% to 40% of the breast cancer cases diagnosed mammographically in the United States of America [2,3].

Currently, it is accepted that DCIS is not one entity but rather a heterogeneous group of lesions with different clinical, radiological, morphological and genetic features [4,5].

Genetic and molecular studies have been published aiming to establish prognostic and predictive factors and new targeted therapies to reduce the risk of recurrence and progression to invasive carcinoma in patients with DCIS [2,6-12]. These advances may become an important part of evaluating DCIS, but at this time, size, grade, comedonecrosis and margin status are established as critical elements in the reporting of DCIS [1,13].

The purpose of this study was to determine the frequencies of DCIS subtypes, nuclear grade and comedonecrosis of a series of cases of DCIS of the breast; to compare the age of patients with the histopathological characteristics of DCIS, and to assess the agreement of grade between in situ and invasive components in DCIS cases that were associated with invasive carcinoma.

## Methods

Four hundred and three cases of DCIS, pure or associated with invasive carcinoma, were consecutively identified from the histopathology files of the Breast Pathology Laboratory, School of Medicine, Federal University of Minas Gerais, Brazil, from 2003 to 2008. Histopathological sections from all cases were reviewed by two authors (HG and AAP) and data considered in the analysis was that obtained in the current slide review.

The criteria defined by World Health Organization (2012) were used for histopathological diagnosis, classification and grading of DCIS and invasive carcinoma [1]. The nuclear grade of DCIS was classified as low, intermediate or high on the basis of nuclear size, pleomorphism, chromatin pattern, presence of nucleoli and mitotic activity. DCIS with low nuclear grade consists of a monotonous population of cells with slightly enlarged nuclei, smooth nuclear membranes, finely dispersed chromatin, inconspicuous nucleoli and rare mitoses. The cells of low-grade DCIS are typically polarized with the longest axis of the cell oriented perpendicularly to the basement membrane, and radially distributed around neoformed extracellular lumina. DCIS of intermediate nuclear grade consists of a population of cells with intermediate-size nuclei with coarser chromatin and evident but still inconspicuous nucleoli. Mitotic activity may be encountered, but it is rarely high. The neoplastic cells may be polarized. DCIS of high nuclear grade consists of cells with large (>2.5 times the size of a red blood cell) and pleomorphic nuclei that show vesicular and coarse chromatin, with prominent and often multiple and irregular nucleoli. The neoplastic epithelial cells usually lack polarity, and mitotic activity is easily detected [1,14]. The highest nuclear grade was used for the purpose of statistical analysis. The nuclear grade of DCIS was not evaluated in eleven cases (2.7%) because the slides were not available for review. The grade of invasive carcinoma was classified as low, intermediate or high based on an assessment of tubule/gland formation, nuclear pleomorphism and mitotic count [1]. Tubular formation was assessed over the whole tumour; nuclear pleomorphism was evaluated in the area showing the highest degree of pleomorphism, and mitotic counting was performed in the area exhibiting most proliferation [1].

The architectural patterns of DCIS included solid, cribriform, micropapillary, papillary and apocrine [1]. DCIS was divided into single (when >90% of the in situ tumor displayed one architectural growth pattern) and mixed (when the dominant pattern constituted <90% of the in situ carcinoma) [15].

The term comedonecrosis, which is poorly defined in the literature, was applied when significant necrosis, creating an appearance similar to comedos, seen in cutaneous acne, was noted in ducts involved by DCIS [15,16].

We measured the largest focus of all pure DCIS cases. Because not all slides from each case were available to be reviewed, we did not analyze margin status and size of DCIS in cases associated with invasive carcinoma.

Pearson’s asymptotic test was used to compare proportions. The t test was used to compare age means among the groups and the Bonferroni test was used to multiple comparisons between them. The weighted kappa test was used to assess the concordance between nuclear grade of DCIS and histological grade of invasive carcinoma. Kappa values in the range 0.21 to 0.40 demonstrated fair agreement [17]. A *p* value <0.05 was considered statistically significant. This study was approved by the Research Ethics Committee of the Federal University of Minas Gerais (protocol ETIC 655/08).

## Results

Pure DCIS was detected in 110/403 cases (27.3% of the total) and 293/403 cases (72.7% of the total) were DCIS associated with invasive carcinoma.

The mean age of patients at diagnosis was 54.1 years (standard deviation ± 13.1). There was no significant difference in age between pure DCIS and DCIS associated with invasive carcinoma (p = 0.814).

The mean size of pure DCIS was 15.2 mm (range: 2 to 100 mm; standard deviation ± 15.8). There was no significant difference between the size of pure DCIS and age (p = 0.938), neither between the size of pure DCIS and presence of comedonecrosis (p = 0.732). We did not find a significant difference in size between single growth pattern and mixed growth pattern (p = 0.213), and also between the size and the nuclear grade (p = 0.175). There was no significant difference between the size and the subtype of DCIS (p = 0.137). However, we identified a tendency of the micropapillary subtype to be larger than the other subtypes (p = 0.06).

The frequencies of DCIS subtypes are shown in Table 1. Of the 403 cases of DCIS (pure and associated with invasive carcinoma), 222 cases (55.1%) displayed a single growth pattern and 181 cases (44.9%) showed a mixed growth pattern. Among architectural patterns, the solid subtype was the most common (170/403 cases; 42.2%). The pure micropapillary subtype was found in 13/403 cases (3.2%). The apocrine morphology was not identified among DCIS with a single architectural pattern. There was no significant difference in single or mixed growth pattern between pure DCIS and DCIS associated with invasive carcinoma (p = 0.088).

**Table 1:** **Frequencies of ductal carcinoma in situ subtypes**

**Architectural pattern**	**N**	**%**
**Solid** *	170	42.2
**Cribriform** *	27	6.7
**Papillary** *	12	3.0
**Micropapillary** *	13	3.2
**Apocrine** *	00	00
**Mixed**	181	44.9
**Total**	403	100

*Single growth pattern.

The nuclear grade of DCIS was evaluated in 392/403 cases (97.3%; Fig. 1A-C). High-grade DCIS was identified in 293/403 cases (72.7%; Figure 1C). There was no significant difference in nuclear grade between pure DCIS and DCIS associated with invasive carcinoma (p = 0.142). The frequencies of different nuclear grades of DCIS and the relationship between nuclear grade and different single architectural patterns are respectively shown in Tables 2 and 3. Among DCIS with a single architectural pattern, high grade was more common in the solid subtype (151/168 cases, 89.9%; p < 0.001). Only 32% of tumors with a cribriform pattern had high nuclear grade.

**Figure 1:** **Ductal carcinoma in situ of the breast: different nuclear grades and comedonecrosis.** **A** - Low grade ductal carcinoma in situ, cribriform type, showing uniform cells with mild atypia. Hematoxylin and eosin, x200. **B** – Intermediate grade ductal carcinoma in situ, showing cells with mild a moderate atypia and focal necrosis. Hematoxylin and eosin, x200. **C** – High grade ductal carcinoma in situ, solid type, showing severe atypical cells, without necrosis. Hematoxylin and eosin, x400. **D** – High grade ductal carcinoma in situ, solid type with extensive comedonecrosis. Hematoxylin and eosin, x200.

**Table 2:** **Frequencies of nuclear grade of ductal carcinoma in situ**

**Nuclear grade**	**N**	**%**
**Low grade**	38	9.4
**Intermediate grade**	61	15.2
**High grade**	293	72.7
**Missing**	11	2.7
**Total**	403	100

**Table 3:** **Nuclear grade and architectural patterns of ductal carcinoma in situ**

			**Architectural**	**Pattern** *	
**Nuclear grade**	**Solid N (%)**	**Cribriform N (%)**	**Papillary N (%)**	**Micropapillary N (%)**	**Total**
**Low**	08 (4.8)	08 (32.0)	02 (16.7)	02 (16.7)	20 (9.2)
**Intermediate**	09 (5.3)	09 (36.0)	01 (8.3)	01 (8.3)	20 (9.2)
**High**	151 (89.9)	08 (32.0)	09 (75.0)	09 (75.0)	177 (81.6)
**Total**	168 (100)	25 (100)	12 (100)	12 (100)	217 (100)
**Missing**	02	02	00	01	p < 0.001

*Single growth pattern; p = significance level.

Comedonecrosis was present in 222/403 cases (55%; Figure 1D). The frequencies of comedonecrosis in different architectural patterns are shown in Table 4. Among DCIS cases with a single growth pattern, comedonecrosis was more often in cases with a solid morphology (p < 0.001). The cribriform, papillary and micropapillary subtypes more frequently did not present comedonecrosis (p < 0.001).

**Table 4:** **Comedonecrosis and architectural patterns of ductal carcinoma in situ**

		**Architectural**		**Pattern** *	
**Comedonecrosis**	**Solid N (%)**	**Cribriform N (%)**	**Papillary N (%)**	**Micropapillary N (%)**	**Total**
**Absent**	36 (21.2)	21 (77.8)	09 (75.0)	08 (61.5)	74 (33.3)
**Present**	134 (78.8)	06 (22.2)	03 (25.0)	05 (38.5)	148 (66.7)
**Total**	170 (100)	27 (100)	12 (100)	13 (100)	222 (100) p < 0.001

*Single growth pattern; p = significance level.

Patients with high-grade DCIS were younger (mean age = 53 years) in relation to patients with low-grade DCIS (mean age = 58.4 years; p = 0.027). Patients with tumours with comedonecrosis were also younger in comparison to patients with tumours without comedonecrosis (p = 0.003).

Invasive carcinoma of no special type was the most common (262/293 cases; 88.7%), followed by the tubular carcinoma (12/293 cases; 4.1%), mucinous carcinoma (07/293 cases; 2.4%), invasive lobular carcinoma (04/293 cases; 1.4%), invasive papillary and micropapillary carcinomas (03/293 cases each one; 1%), secretory and cribriform carcinomas (02/293 cases each one; 0.7%).

Fair agreement was observed between in situ and invasive components with regard to grade (weighted kappa = 0.23).

## Discussion

In the present study we evaluated morphological features of a series of DCIS pure (110 cases, 27.3% of the total) or associated with an invasive component (293 cases, 72.7% of the total) correlating them with the age of patients. Clinical and histological characteristics that may predict the risk of recurrence in women with DCIS include the age, tumour grade, presence of comedonecrosis, architectural subtype, tumour size, and width of resection margin [18,19]. In our series we evaluated nuclear grade, tumour size, comedonecrosis and age that are well established critical elements in the reporting of DCIS. Although recent genetic, molecular and immunohistochemical studies have contributed to advances in the understanding of the pathogenesis of DCIS, age and histopathological features remain the most established predictors of behavior in DCIS [1,8,20-26].

In our series, the majority of the cases (293 cases, 72.7% of the total) were high-grade DCIS; 15.2% of cases had an intermediate grade and 9.4% were low-grade CDIS. The classification of DCIS has been based on the architectural growth pattern. Cytonuclear differentiation of tumour cells is more important than the architectural growth pattern and various novel classifications of DCIS have been proposed. Almost all modern classifications separate DCIS into three categories (high, intermediate, and low grade), but differ in the choice of features that are used for categorization [27]. Studies have reported nuclear grade to be the most significant predictor of recurrence on both univariate and multivariate analysis [28,29]. Therefore, cytonuclear grade has been used as the basic method for the assessment of intrinsic biological aggressiveness. Scripcaru and colleagues recognized, respectively, high-grade DCIS and intermediate nuclear grade in 45% and 41% of their cases [15]. These differences in the frequencies of grade are possibly attributed to the variation in the classification criteria, to the differences between the populations or to the detection method of the tumours (clinical or mammographically detected tumours).

We also correlated the nuclear grade of DCIS with the histological grade of invasive carcinoma to assess the agreement between in situ and invasive components in DCIS cases that were associated with invasive carcinoma. The fair agreement between in situ and invasive components with regard to grade (weighted kappa = 0.23) observed in our study is probably related to the various categories (grades 1, 2 or 3) included in the statistical analysis.

We showed that comedonecrosis was significantly more often in solid morphology than in cribriform, papillary and micropapillary subtype (p < 0.001). Scripcaru et al. also identified a statistically significant difference between the presence of comedonecrosis in micropapillary and solid subtypes versus the cribriform morphology [15]. Comedonecrosis may be seen in association with any architectural pattern. The term “comedo DCIS” is widely used in historical series but does not confer either a specific grade or architecture to the lesion and there is no consensus in the literature regarding the amount of central necrosis required, so reproducibility as a category of DCIS is questionable [4]. Although rates of ipsilateral breast tumour recurrence are generally higher for tumours with a component of comedonecrosis than for those without, irrespective of adjuvant therapies, the presence of necrosis might be a weaker predictor of ipsilateral breast tumor recurrence than cellular architecture and nuclear grade [30].

The architectural patterns of DCIS include solid, cribriform, micropapillary, papillary and unusual variants (apocrine, signet ring, neuroendocrine, spindled, squamous or clear cells) [1]. Some combinations of nuclear grade and architectural pattern tend to be more frequent than others but any combination can occur [7]. The current World Health Organization classification does not recognize the low-grade (monomorphic) variant of DCIS with an exclusive flat type (clinging) pattern and did not recommend this terminology [1].

Our results showed that high grade was more common in the solid subtype (89.9%; p < 0.001) and only 32% of tumors with a cribriform pattern had high nuclear grade. Solid DCIS is characterized by a proliferation of neoplastic cells that fill, expand, and distort a duct. Nuclear grades can range from high to low in solid DCIS, although pure solid DCIS with low nuclear grade is fairly rare. Low-grade DCIS with solid architecture sometimes raises the differential diagnosis of lobular carcinoma in situ [1,31-33]. Cribriform DCIS is characterized by well-defined lumens lined by neoplastic cells. Such an orderly arrangement is rare in high-grade DCIS [7].

DCIS most frequently (62%) shows a mixture of architectures, which is seen almost twice as often as the second most commonly seen pattern (solid, 31.9%) [4]. In our series, 55.1% of cases displayed a single growth pattern and 44.9% showed a mixed growth pattern. Among architectural patterns, the solid subtype was more common (42.2%). Similar to our results, Scripcaru and colleagues also described that 58% of cases of DCIS displayed a single growth pattern and 42% showed a mixed growth pattern [15].

Silverstein’s group showed age to be an independent prognostic factor for local recurrence, which led to incorporation of age into the Van Nuys Prognostic Index by the division of patients into three groups (≥ 61 years, 40–60 years and ≤ 39 years) [34]. Goldstein et al. examined pathologic features of DCIS in three different age groups of patients to identify differences that might explain why young patient age at the time of diagnosis is a risk for recurrence. They found that younger patients more frequently had higher nuclear grade DCIS, central necrosis, smaller initial biopsy maximum dimensions and close or positive margins [35].

In our series, patients with high grade DCIS were younger in relation to patients with low grade DCIS (p = 0.027) and patients with tumours with comedonecrosis were also younger in comparison to patients with tumours without comedonecrosis (p = 0.003). This group of younger patients may have an increased risk of local recurrence when treated with breast-conserving therapy due to a greater proportion of high nuclear grade DCIS and presence of comedonecrosis. In the present study, the type of treatment (radical or breast-conserving therapy) and the local recurrence were not evaluated. Maybe the association of high nuclear grade DCIS, comedonecrosis and younger patients can guide the clinicians to perform more aggressive surgical treatments, as these factors are associated with local recurrence.

## Conclusions

The high nuclear grade and the presence of comedonecrosis were identified more frequently in DCIS of younger patients and more often correlated with the solid pattern DCIS. As clinical and histopathological features remain the most established predicts of behavior in DCIS, the choice of surgical treatment should be guide by them in addition to the size of DCIS and margin status.

### Consent

Written informed consent was obtained from the patients for the publication of this report and any accompanying images.

## Abbreviation

DCIS: Ductal carcinoma in situ
